# A Self-Representation-Based Fuzzy SVM Model for Predicting Vascular Calcification of Hemodialysis Patients

**DOI:** 10.1155/2021/2464821

**Published:** 2021-07-27

**Authors:** Xiaobin Liu, Xiran Zhang, Xiaoyi Guo, Yijie Ding, Weiwei Shan, Liang Wang, Wei Zhou, Hua Shi

**Affiliations:** ^1^Department of Nephrology, The Affiliated Wuxi People's Hospital of Nanjing Medical University, 214023, Wuxi, China; ^2^School of Electronic and Information Engineering, Suzhou University of Science and Technology, 215009, Suzhou, China; ^3^School of Opto-Electronic and Communication Engineering, Xiamen University of Technology, 365001, Xiamen, China

## Abstract

In end-stage renal disease (ESRD), vascular calcification risk factors are essential for the survival of hemodialysis patients. To effectively assess the level of vascular calcification, the machine learning algorithm can be used to predict the vascular calcification risk in ESRD patients. As the amount of collected data is unbalanced under different risk levels, it has an influence on the classification task. So, an effective fuzzy support vector machine based on self-representation (FSVM-SR) is proposed to predict vascular calcification risk in this work. In addition, our method is also compared with other conventional machine learning methods, and the results show that our method can better complete the classification task of the vascular calcification risk.

## 1. Introduction

Cronic kidney disease-mineral bone disease (CKD-MBD) is one of the most serious complications in patients with end-stage renal failure, including an abnormal metabolism of calcium, phosphorus, parathyroid hormone, vitamin D, abnormal bone transformation, vascular calcification, and ultimately cardiovascular disease.

In recent years, fibroblast growth factor (FGF23) has been recognized as a protein that plays an important role in phosphate regulation. Klotho protein is the receptor protein of FGF23. It participates in regulating the body's bone metabolism, calcium and phosphorus metabolism, protecting the integrity of blood vessels, and inhibiting vascular calcification through the formation of FGF23-klotho complexes. Therefore, FGF23 and klotho are key participants in CKD-MBD, and they are closely related to the occurrence of vascular calcification and cardiovascular disease. Existing evidence shows that there is a clear correlation between FGF23 and the occurrence of vascular calcification and cardiovascular disease (CVD). The increase of FGF23 can be used as a risk factor for CVD in patients with end-stage renal disease (ESRD) [1].

Fetuin-A is considered to be an inhibitor of the progression of vascular calcification and can delay the progression of abdominal aortic calcification [2]. Studies have shown that there is a close correlation between fetuin-A and the malnutrition-microinflammatory state of ESRD patients [2]. It is currently believed that low serum fetuin-A levels in ESRD patients is an independent risk factor for vascular calcification.

Malnutrition is a common complication in ESRD patients, and it is closely related to vascular calcification, cardiovascular events, and all-cause mortality. Factors affecting the nutrition of ESRD patients include protein-energy expenditure, digestion and absorption, inflammation, and endocrine hormone level disorders [3].

There are a variety of tools available to assess the nutritional status of dialysis patients. Among them, the geriatric nutrition risk index (GNRI) is considered to be an important predictor of cardiovascular death [4]. The latest research also shows that there is a certain positive correlation between GNRI and the degree of aortic calcification in CKD patients [5].

Vascular calcification (VC) scores of the artery or aorta on plain radiographs are associated with CVD events and may be predictive of CVD in dialysis patients [6]. Many research results show that abdominal aortic calcification as assessed on a lateral lumbar X-ray is predictive for the presence of significant coronary artery disease in asymptomatic dialysis patients [7].

The previous research results of our work show that patients with end-stage renal failure have abnormal levels of FGF23 and klotho and microinflammatory states. Their interaction and mutual influence are involved in the occurrence and development of vascular calcification and CKD-MBD [8].

Therefore, in order to further explore the risk factors of vascular calcification in patients with ESRD, this article studies the scientific and accurate prediction of vascular calcification risk factors in ESRD patients with different forecasting model, so as to help clinicians to detect and intervene early, thereby delaying the occurrence and development of CKD-MBD, reducing the incidence of CVD, and improving the prognosis. Machine learning (ML) has been widely used in the dry weight (DW) [9] of hemodialysis patients and has achieved good results. Lots of ML-based models also have been well used in drug discovery [10–12], protein function [13–16], and disease analysis [17, 18].

In this study, we employ a support vector machine (SVM) to build a predictive model. SVM has the following advantages: (1) Nonlinear mapping is the theoretical basis of the SVM method. SVM uses the inner product kernel function to replace the nonlinear mapping to high-dimensional space. (2) The optimal hyperplane to divide the feature space is the goal of SVM, and the idea of maximizing the classification margin is the core of the SVM method. (3) A small number of support vectors determine the final result, which can not only help us capture key samples but also “remove” a large number of redundant samples. For imbalanced datasets, the standard SVM is not good at classifying a small number of categories. In this work, we propose a fuzzy support vector machine based on self-representation (FSVM-SR) to identify vascular calcification of hemodialysis patients under imbalanced data. FSVM can estimate a weight for each training sample. When constructing the hyperplane of classification, FSVM avoids some low-weight samples (noise samples) to alleviate the influences of imbalanced datasets.

## 2. Materials and Methods

### 2.1. Materials

This work employs 29 features to describe the patient's information, which includes gender, age, body mass index (BMI), diabetes mellitus (DM), cerebral infarction (CI), and coronary heart disease (CHD).  Table 1 shows the details of our dataset. The mean and standard deviation of samples is also list in it.

During the data collection process, we classified 59 patients into risk levels. We roughly classify the 7 risks according to two classification methods. Some adjacent levels will be grouped into one category. The classification results are shown in Table 2. In the first classification scheme (CS1), levels {0, 1, 2} and levels {3, 4, 5, 6} are classified into classes 1 and 2, respectively. In addition, the levels {0, 1}, {2, 3}, and {4, 5, 6} are classified into classes 1, 2, and 3 (in CS2), respectively.

### 2.2. Methods

#### 2.2.1. Abdominal Aortic Calcification

All patients need to undergo lateral lumbar X-ray examination within 1 week of blood biochemical examination to assess the calcification of the abdominal aorta corresponding to levels 1-4 [7]. According to the length of the calcified plaques on the anterior and posterior walls of the abdominal aorta, for scores of 0 to 3: no calcification is 0 points, calcification range<1/3 arterial wall length is 1, calcification range 1/3-2/3 arterial wall length is 2, calcification range>2/3 arterial wall length is 3, and total score is between 0 and 24. Two radiologists separately scored and averaged. The calculation of geriatric nutrition risk index (GNRI) [19] can be estimate by

(1) $$\begin{array}{c} \text{GNRI}=\left[14.89\times \text{serum albumin}\right]+\left[41.7+\left(\frac{\text{actual body weight}}{\text{ideal body weight}}\right)\right]. \end{array}$$

Serum levels of intact FGF23, soluble Klotho, Fetuin-A, and interleukin-6 were received by using two-site enzyme-linked immune assays (reagents from Elabscience Biotech, Wuhan, China).

#### 2.2.2. Fuzzy Support Vector Machine

SVM is a robust machine learning method based on statistical learning, which considers empirical risk and adds a regularization term to reduce structural risk. It is a sparse and robust classifier [20]. SVM also can perform nonlinear classification through the kernel method, which is one of the common kernel learning methods. In many practical classification tasks, the number of samples in different categories is often different. Under the imbalanced dataset, the SVM model will produce a large deviation. In order to avoid the above situation, Lin and Wang proposed fuzzy SVM (FSVM) [21]. Different from SVM, FSVM uses membership value to describe the weight of the training sample. In general, the membership value of outlier samples is lower, and it is easier for the algorithm to weaken the contribution to the decision hyperplane during the training process.

For FSVM, a training sample can be defined as {**x**_*i*_, *y*_*i*_, *s*_*i*_}, *i* = 1, 2, ⋯, *N*, where *N* is the number of training samples, **x**_*i*_ ∈ R^*d*×1^, *y*_*i*_ and *s*_*i*_ ∈ [0, 1] are feature vector, label, and membership value of sample *i*, respectively. The feature vector dimension of the model is *d*. The objective optimization function of FSVM is

(2) $$\begin{array}{c} \begin{array}{c} \min\frac{1}{2}{\left\|w\right\|}^{2}+C\overset{N}{\underset{i=1}{\sum }}s_{i}\xi_{i},\\ s.t.y_{i}\left(w^{T}\phi \left(x_{i}\right)+b\right)\geq 1-\xi_{i},\\ \;\xi_{i}\geq 0,i=1,2,\cdots ,N, \end{array} \end{array}$$

where *C* denotes the regularization parameter, *ξ*_*i*_ is the error measure of **x**_*i*_. To build a robust model, different training samples should be given different regularization parameters. *s*_*i*_*ξ*_*i*_ is the error measure, which is weighted by the membership value. Outliers (noise) have a lower weight; on the contrary, important sample points will have a higher weight. In an imbalanced dataset, the type of data with a large number of samples often contains more outliers. In order to reduce the deviation, FSVM can well reduce its impact. Equation (2) also can be rewritten by the Lagrange dual problem:

(3) $$\begin{array}{c} \begin{array}{c} \max\overset{N}{\underset{i=1}{\sum }}\alpha_{i}-\frac{1}{2}\overset{N}{\underset{i=1}{\sum }}\overset{N}{\underset{j=1}{\sum }}\alpha_{i}\alpha_{j}\cdot y_{i}y_{j}\cdot K\left(x_{i},x_{j}\right),\\ s.t.\;0\leq \alpha_{i}\leq s_{i}C,\\ \;\overset{N}{\underset{i=1}{\sum }}\alpha_{i}y_{i}=0,\;i=1,2,\cdots ,N, \end{array} \end{array}$$

where *α*_*i*_ is the Lagrange multiplier coefficient for sample **x**_*i*_. *K*(**x**_*i*_, **x**_*j*_) is the value of samples *i* and *j* in the kernel matrix. And the kernel matrix can be calculated by the radial basis function (RBF):

(4) $$\begin{array}{c} \begin{array}{c} K\left(x_{i},x_{j}\right)=\exp\left(-\gamma {\left\|x_{i}-x_{j}\right\|}^{2}\right),\\ \;i,j=1,2,\cdots ,N, \end{array} \end{array}$$

where *γ* is a Gaussian kernel bandwidth.

The final decision function of classification is

(5) $$\begin{array}{c} f\left(x\right)=\mathrm{sign}\left[\overset{N}{\underset{i=1}{\sum }}y_{i}\alpha_{i}\cdot K\left(x,x_{i}\right)+b\right]. \end{array}$$

The basic SVM can only perform binary classification tasks. In this work, we use the one-against-one strategy to achieve multiple classifications.

#### 2.2.3. Self-Representation-Based Membership Function

In this work, we propose a method based on a reconstruction error to construct the membership function. This method can measure the consistency between the overall data structure and a single data point. The reconstruction error can quantify the outlier degree of the noise sample, which helps to improve the robustness of the model.

Let **X** = {**x**_1_, **x**_2_, ⋯, **x**_*N*_} ∈ **R**^*d*×*N*^, the self-representation function is defined as follows:

(6) $$\begin{array}{c} X=XZ+E, \end{array}$$

where **Z** = [**z**_1_, **z**_2_, ⋯, **z**_*N*_] ∈ **R**^*N*×*N*^ and **E** ∈ **R**^*d*×*N*^ are the coefficient and error matrix. **z**_*i*_ is the new representation of sample *i* by other training samples. The self-representation formulation can be optimized by

(7) $$\begin{array}{c} \min\;J\left(Z\right)={\left\|XZ-X\right\|}_{F}^{2}+\lambda Tr\left({ZLZ}^{T}\right), \end{array}$$

where *Tr*(**ZLZ**^*T*^) is the Laplacian regular term to smooth the coefficient **Z**:

(8) $$\begin{array}{c} Tr\left({ZLZ}^{T}\right)=\frac{1}{2}\overset{N}{\underset{i=1}{\sum }}\overset{N}{\underset{i=1}{\sum }}W_{ij}{\left\|z_{i}-z_{j}\right\|}_{2}^{2}, \end{array}$$

where **W** is the similarity matrix between samples. It also can be replaced by kernel matrix. **L** = **D**^−1/2^Δ**D**^−1/2^ is a normalized Laplacian matrix and Δ = **D** − **W**. The *D*_*ii*_ = ∑_*j*=1_^*N*^*W*_*ij*_ is an element of the diagonal matrix **D** ∈ **R**^*N*×*N*^. In this work, *λ* denotes the coefficient of the Laplacian regular term, which is set as 0.01. Setting *∂J*(**Z**)/*∂ ***Z** = 0, the solution of Equation (7) can be obtained as follows:

(9) $$\begin{array}{c} \begin{array}{c} \frac{\partial J\left(Z\right)}{\partial Z}=0,\\ 2X^{T}\left(XZ-X\right)+2\lambda ZL=0,\\ X^{T}XZ+\lambda ZL=X^{T}X, \end{array} \end{array}$$

where **X**^*T*^**XZ** + *λ ***ZL** = **X**^*T*^**X** is a Sylvester equation. For each training sample, the reconstruction error of **x**_*i*_ can be calculated as

(10) $$\begin{array}{c} r_{i}={\left\|{Xz}_{i}-x_{i}\right\|}_{2}^{2}. \end{array}$$

To map the value of reconstruction error in 0 ~ 1. We define the following formula:

(11) $$\begin{array}{c} s_{i}=1-\frac{r_{i}-r_{\min}}{r_{\max}-r_{\min}}, \end{array}$$

where *r*_min_ and *r*_max_ are the minimum and maximum reconstruction errors, respectively. The process of our method is list in Algorithm 1.

## 3. Results

### 3.1. Evaluation measurements.

In our study, the accuracy (ACC) is employed to evaluate the predictive performance of our predictive model. In addition, a 10-fold crossvalidation method [22–25] was used in this work. The calculation method of ACC is as follows:

(12) $$\begin{array}{c} \text{Whole ACC}=\frac{\sum_{i=1}^{c}{\text{TP}}^{i}}{M}\times 100\%,\\ {\text{ACC}}^{i}=\frac{{\text{TP}}^{i}}{M^{i}}\times 100\%,\\ M=\overset{c}{\underset{i=1}{\sum }}M^{i}, \end{array}$$

where TP^*i*^ is the number true positive (TP) in subclass *i*. *c* is the number of classes. *M* and *M*^*i*^ denote the number of whole test samples and subclass test samples. ACC^*i*^ is the accuracy of subclass *i*.

## 4. Selection of Optimal Parameters

In order to obtain the best prediction performance, we use the grid search method to obtain the optimal parameters *C* and *γ*. The search ranges are from 2^−5^ to 2^10^ (*C*), and from 2^−10^ to 2^5^ (*γ*), with the step of 2^1^. Figures 1.  and 2 show the average ACC with different *C* and *γ* (under CS1 and CS2), respectively.

As shown in the figures, the model reach ACC of 83.05% and 64.40%, when the optimal parameters *C* = 27, *γ* = 2^−6^and *C* = 210, *γ* = 2^−6^, respectively.

### 4.1. Comparison to Other Classifiers

To further evaluate the performance of our model, we introduced other similar machine learning models [26, 27], including logistic regression, back propagation (BP) neural network, radial basis function (RBF) neural network, Takagi-Sugeno-Kang fuzzy system (TSK-FS) [28–30], and standard SVM. Under 2 classes (Table 3), logistic regression, BP network, RBF network, and TSK-FS achieve whole ACC of 71.18%, 66.10%, 77.96%, and 76.27%, respectively. The whole ACC of SVM (79.66%) and FSVM-SR (83.05%) are better than other models. In particular, FSVM-SR obtains the best prediction accuracy. In subclasses 1 and 2, FSVM-SR also achieves best accuracy of 95.23% and 52.94%, respectively. It can be seen from the results that for small sample learning, the SVM has more advantages than the neural network models. As the fuzzy model, FSVM has better performance than TSK-FS on this dataset. FSVM-SR can effectively suppress the influence of noise samples on the model. The receiver operating characteristic curves (ROC) of different models are shown in Figure 3. It can also be found that our method obtains the highest area under curve (AUC) value of 0.7955.

Under CS3, FSVM-SR also compares with these predictors, and the results of comparison are listed in Table 4. SVM and FSVM-SR achieve the best whole ACC of 64.40%. In subclass 1, the ACC of RBF neural network and SVM are 72.00% (best). FSVM-SR and TSK-FS obtain 65.21%, and FSVM-SR has smaller standard deviation (30.88%) in subclass 2. In addition, SVM and FSVM-SR have better performance (54.54%) in subclass 3. It can be seen that FSVM-SR is also more stable and effective in the case of CS3.

Two-sample *t*-test is employed to evaluate the significance differences of average ACC value in CS1 and CS2, respectively. In our work, the significance level is 0.05. FSVM-SR is compared with other models via 10-fold crossvalidation (20 times). The results of statistical significance are shown in Table 5. In CS1, the differences between FSVM-SR and other models are all significant (*P* value < 0.05). The max value is 0.0064 (for SVM) and min value is 3.4341*e*-11 (for BP neural network). Except for SVM (*P* value 0.1965), the differences with other models are significant in CS2. It can be seen from the results that the proposed method (FSVM-SR) outperforms most methods in two patient risk classification schemes.

## 5. Discussion

Cardiovascular death is the main cause of ESRD patients. Studies have confirmed that the occurrence of abdominal aortic calcification (in ESRD patients) is extremely important for cardiovascular death [31]. In recent years, the influence of nontraditional risk factors, such as FGF23, klotho abnormality, microinflammatory state, and malnutrition on vascular calcification has attracted much attention from scholars.

As a protein that plays a key role in phosphate regulation, FGF23 is involved in controlling the metabolism of phosphate, parathyroid hormone, and 1,25 dihydroxy vitamin D. FGF23 can not only regulate phosphate homeostasis but also further promote disease progression, left ventricular hypertrophy, and increase the occurrence and death of CVD [1]. Klotho, as an antiaging gene, has been confirmed by many studies that it participates in cardiovascular protection in ESRD patients by inhibiting phosphate-driven vascular calcification [32]. The results of previous studies of our center showed that serum FGF23 levels increased, and soluble klotho levels decreased. Moreover, after the combined abdominal aortic sclerosis, the abnormalities of serum FGF23 and klotho are more obvious [8]. This study is consistent with the results of previous studies. The levels of FGF23 and klotho are abnormal in ESRD patients. They are risk factors for vascular calcification. And the analysis results of different risk prediction models all support this conclusion.

Fetuin-A, as a protective factor for vascular calcification, can inhibit the process of vascular calcification [33]. The results of this study show that the serum fetuin-A of ESRD patients is significantly reduced. In addition, the serum fetuin-A decreases more significantly in patients with abdominal aortic calcification. The level of decrease has a certain early warning effect on vascular calcification. Both FSVM and traditional prediction models suggest that fetuin-A is an independent risk factor for abdominal aortic calcification. Therefore, clinicians should pay close attention to serum fetuin-A levels in the process of CKD. Once abnormalities occur, they should intervene as soon as possible.

Studies have shown that malnutrition is closely related to vascular calcification, cardiovascular death, and all-cause death in ESRD patients [4]. In this work, the results of different risk prediction models support that malnutrition is an independent risk factor for abdominal aortic calcification. Existing studies have shown that malnutrition and microinflammatory state, insulin resistance, FGF23/klotho axis abnormalities, and other factors are interconnected and ultimately jointly promote the occurrence of vascular calcification [19]. Therefore, many risk factors for vascular calcification are often mixed, and it is difficult for clinicians to accurately determine the main risk factors and provide precise treatment intervention. By comparing the accuracy of different prediction models for predicting the risk of abdominal aortic calcification, it is found that the FSVM and SVM models are more accurate in identifying the main risk factors than the traditional logistic regression model. Under CS2, FSVM-SR achieves best accuracy of 95.23% and 52.94%, respectively. Our method (FSVM-SR) is significantly better than other methods (*P* value, logistic regression: 8.4386*e* − 10, BP network: 3.4341*e* − 11, RBF network: 7.9770*e* − 06, TSK-FS: 3.3813*e* − 08, and SVM: 0.0064). What is more, FSVM-SR and SVM achieve the best whole ACC of 64.40% in CS3. Self-representation-based membership function can estimate weight for training sample. The reconstruction error of outliers is relatively large, and the corresponding membership value is low. When constructing the hyperplane of classification, FSVM avoids some low-weight samples (outliers) to alleviate the influences of imbalanced datasets. The fuzzy methods [34] improve the interpretability and robustness of the model. There are related applications in the medical fields [35, 36].

## 6. Conclusions

In this work, we propose a FSVM based on a self- representation method to filter noise samples, improve the generalization ability of the model, and obtain good results. Although our method has achieved a better accuracy, it still has the following disadvantage: (1) The sample size needs to be further increased to minimize the prediction bias. (2) There is no detailed analysis of the various factors of the patient [37, 38]. (3) The interpretability of the model is not as good as that of the linear model. Based on the above, we will propose a sparse linear model in the next work to solve the problem of poor interpretability and factor analysis.

## Figures and Tables

**Figure 1:** The average ACC with different *C* and *γ* (under CS1).

**Figure 2:** The average ACC with different *C* and *γ* (under CS2).

**Figure 3:** The ROCs for different models (under CS2).

**Algorithm 1:** Algorithm of FSVM-SR.

**Table 1:** The information of dataset.

No.	Feature	Value	*r* ^∗^
1	Gender (males/females)	32/27	-0.0455
2	Age (years)	55.83 ± 15.60	0.4010
3	Smoking (yes/no)	1/58	-0.0847
4	BMI (kg/m^2^)	23.56 ± 3.12	0.1639
5	DM (yes/no)	24/35	0.4847
6	CI (yes/no)	3/56	0.0025
7	CHD (yes/no)	5/54	0.0433
8	Systolic blood pressure (mmHg)	155.69 ± 23.63	-0.1150
9	Diastolic blood pressure (mmHg)	88.11 ± 13.71	-0.2043
10	Phosphate binder (yes/no)	36/23	-0.2141
11	Hemoglobin (g/L)	85.38 ± 18.12	-0.2584
12	C-reactive protein (mg/L)	11.74 ± 35.61	0.3016
13	Serum creatinine (*μ*mol/L)	785.09 ± 368.62	-0.4252
14	Serum glucose (mmol/L)	5.48 ± 2.28	0.2608
15	Serum calcium (mmol/L)	2.08 ± 0.24	0.0520
16	Serum phosphorus (mmol/L)	1.81 ± 0.38	-0.0862
17	Total glyceride (mmol/L)	1.69 ± 1.08	-0.0542
18	Total cholesterol (mmol/L)	4.53 ± 1.42	-0.0466
19	Low-density lipoprotein-C (mmol/L)	2.45 ± 0.96	-0.0252
20	High-density lipoprotein-C (mmol/L)	0.97 ± 0.55	0.0866
21	HbA1c (%)	5.82 ± 1.03	0.2151
22	Serum albumin (g/L)	34.31 ± 6.61	-0.1308
23	25-OH vitamin D3 (ng/mL)	7.86 ± 4.55	0.3850
24	iPTH (pg/mL)	274.50 ± 306.31	-0.0225
25	GNRI	96.06 ± 12.76	-0.0078
26	FGF-23 (pg/mL)	32.21 ± 53.02	-0.0966
27	Klotho (ng/mL)	2.38 ± 2.33	0.0443
28	Interleukin-6 (pg/mL)	25.37 ± 53.69	0.2634
29	Fetuin-A (pg/mL)	3.0320e + 05 ± 2.0606e + 05	-0.0234

^∗^Denotes that each feature correlated with ascular calcification level using the Pearson correlation coefficient (*r*).

**Table 2:** The information of patient risk classification scheme.

Risk level	Number of patients	CS1	CS2
0	10	Levels 0, 1, and 2 are class 1 (42 samples)	Levels 0 and 1 are class 1 (25 samples)
1	15		
2	17		Levels 2 and 3 are class 2 (23 samples)
3	6	Levels 3, 4, 5, and 6 are class 2 (17 samples)	
4	6		Levels 4, 5, and 6 are class 3 (11 samples)
5	4		
6	1		

CS: classification scheme.

**Table 3:** Comparison on existing models via 10-fold crossvalidation (under 2 classes).

Model	Whole ACC (%)	ACC^1^ (%)	ACC^2^ (%)
Logistic regression	71.18 ± 15.14	83.33 ± 19.01	41.17 ± 33.75
BP neural network	66.10 ± 13.70	73.80 ± 26.78	47.05 ± 43.78
RBF neural network	77.96 ± 8.67	88.09 ± 15.47	52.94 ± 36.89
TSK-FS	76.27 ± 15.31	85.71 ± 15.42	52.94 ± 43.78
SVM	79.66 ± 10.40	90.47 ± 14.15	52.94 ± 36.89
FSVM-SR (our method)	83.05 ± 9.71	95.23 ± 10.54	52.94 ± 36.89

ACC^1^: the accuracy of class 1; ACC^2^: the accuracy of class 2.

**Table 4:** Comparison on existing models via 10-fold crossvalidation (under 3 classes).

Model	Whole ACC (%)	ACC^1^ (%)	ACC^2^ (%)	ACC^3^ (%)
Logistic regression	57.62 ± 15.25	64.00 ± 32.20	60.86 ± 32.58	36.36 ± 48.30
BP neural network	55.93 ± 19.62	60.00 ± 32.44	60.86 ± 28.60	36.36 ± 47.43
RBF neural network	59.32 ± 21.99	72.00 ± 29.61	60.86 ± 41.91	27.27 ± 48.30
TSK-FS	62.71 ± 24.21	68.00 ± 28.81	65.21 ± 39.13	45.45 ± 49.72
SVM	64.40 ± 17.39	72.00 ± 21.94	60.86 ± 32.44	54.54 ± 49.72
FSVM-SR (our method)	64.40 ± 17.39	68.00 ± 24.85	65.21 ± 30.88	54.54 ± 49.72

ACC^1^: the accuracy of class 1; ACC^2^: the accuracy of class 2; ACC^3^: the accuracy of class 3.

**Table 5:** Analysis of statistical significance for different methods via 10-fold crossvalidation (20 times).

Model	CS1 (*P* value)	CS2 (*P* value)
Logistic regression	8.4386*e* − 10	1.1262*e* − 05
BP neural network	3.4341*e* − 11	6.9318*e* − 07
RBF neural network	7.9770*e* − 06	0.0013
TSK-FS	3.3813*e* − 08	0.0024
SVM	0.0064	0.1965

## Data Availability

The data used to support the research can be obtained from the corresponding authors according to the requirements of the institution.
